The article "Glucocorticoids Should Be Used With Caution in Patients With SARS-CoV-2" was retracted in 2022. Reason: duplicate publication.

# Glucocorticoids Should Be Used With Caution in Patients With SARS-CoV-2

**DOI:** 10.3389/fmed.2021.564943

**Published:** 2021-02-24

**Authors:** Yong Guo, Yan Chen, Yingchuan Li

**Affiliations:** ^1^Department of Critical Care Medicine, Shanghai Jiao Tong University Affiliated Sixth People's Hospital, Shanghai, China; ^2^Department of Clinical Pharmocology, Shanghai Jiao Tong University Affiliated Sixth People's Hospital, Shanghai, China; ^3^Department of Critical Care Medicine, Shanghai Public Health Clinical Center, Fudan University, Shanghai, China

**Keywords:** glucocorticoid, COVID-19, SARS-CoV-2, pneumonia, inflammation

## Abstract

Severe acute respiratory syndrome coronavirus 2 (SARS-CoV-2) has become a global pandemic, and the use of glucocorticoids in clinical practice is controversial. Our clinical experiences with glucocorticoid treatment suggested that, while use was effective in some cases, in other cases, glucocorticoid were ineffective and even resulted in immunosuppression that could lead to deterioration. Therefore, glucocorticoids should be used with caution in patients with SARS-CoV-2.

## Introduction

On December 31, 2019, a new type of coronavirus disease (SARS-CoV-2) was first reported in Wuhan, Hubei Province, and subsequently, a rapid epidemic was reported in China. However, while SARS-CoV-2 is a new type of infectious pneumonia that threatens patients' lives, medical staff, and scientific researchers lack a clear understanding of the pathophysiological process of severe new coronavirus pneumonia; however, diagnosis, and treatment experience is also accumulating. Therefore, clinical treatments have been based on previous experiences. Previous conventional treatments used for severe acute respiratory syndrome (SARS), influenza virus pneumonia, acute respiratory distress syndrome (ARDS), and other severe diseases include oxygen therapy, respiratory assistance therapy, extracorporeal membrane oxygenation (ECMO) life support, infection control, and nutritional support, but there is a lack of drugs with precise therapeutic effects (including antiviral drugs). The use of glucocorticoids in clinical practice is also controversial (1, 2).

## Clinical Controversy in the Use of Glucocorticoids in Severe Viral Pneumonia

During the acute phase of ARDS, alveolar injury is accompanied by a large number of inflammatory cell infiltrations, macrophage activation, and the release of a large number of inflammatory mediators. Early emergence of alveolar epithelial-mesenchyme transition and initiation of fibrosis are the pathophysiological basis of hormone-assisted therapy. Corticosteroids have potential advantages in the treatment of patients with ARDS because they can regulate the inflammatory response and slow the fibrosis process. However, the results of previous clinical studies based on SARS or severe influenza pneumonia are inconsistent about whether glucocorticoids improve patient outcomes. A clinical observational study on severe H7N9 influenza virus pneumonia showed that treatment with glucocorticoids (equivalent to methylprednisolone 80 mg/day; quartile range, 40–120 mg/day) for 7 days significantly increased the 60-day mortality of patients. In addition, high-dose glucocorticoids (equivalent to methylprednisolone > 150 mg/day) significantly increased the 30- and 60-day mortality and delayed virus clearance (3). Among 309 patients with severe Middle East respiratory distress syndrome (MERS), ICU mortality and hospital mortality increased significantly in patients treated with glucocorticoids, and 90-day mortality in patients treated with glucocorticoids was not significantly different from that in patients without hormone treatments, but virus clearance was delayed (4). The results of a propensity score matching study involving 1,846 patients with severe influenza pneumonia showed that combined hormone therapy (equivalent to methylprednisolone 80 mg/day; quartile range, 60–120 mg/day) was associated with increased ICU mortality (5). A retrospective analysis of a small sample of 78 severely ill patients with SARS showed that hormone therapy could increase the chances of ICU admission or mortality by 20.7 times (6). Studies have also shown that early application of hormone therapy could increase plasma virus load and delay virus clearance (7). Therefore, scholars believe that the application of glucocorticoids for severe new coronavirus pneumonia will not benefit patients and may even be harmful; however, most of the above studies were observational or retrospective studies with selective bias and confounding factors, which might lead to the conclusion that hormone therapy was harmful and the evidence was insufficient. A retrospective analysis of a larger sample (401 cases) of patients with SARS showed that the combined use of hormone therapy did not benefit patients, but the application of hormones (methylprednisolone 133.5 ± 102.3 mg/day) in severe patients (152 cases) could shorten the length of hospital stay and reduce all-cause mortality (8). A prospective cohort study of 2,141 patients with H1N1 influenza virus pneumonia showed that low to moderate doses of glucocorticoids (equivalent to methylprednisolone 25–150 mg/day) could reduce mortality in patients with an oxygenation index below 300 mmHg (9). In addition, a systematic review showed that glucocorticoid therapy in severe community-acquired pneumonia can reduce patient mortality, shorten the duration of mechanical ventilation, and help to prevent ARDS (10).

## Clinical Status of Glucocorticoid Application in New Coronavirus Pneumonia

The summary description of limited autopsy and puncture tissue pathology in the seventh edition of the “New Coronavirus Diagnosis and Treatment Program” shows that serous fluid, fibrin exudate, and transparent membrane formation are observed in the alveolar cavity, and the exudative cells are mainly monocytes and macrophages. The alveolar septum is hyperaemic and oedematous with infiltration of monocytes and lymphocytes. Degeneration and necrosis can be seen in cardiomyocytes, and infiltration of lymphocytes, monocytes, and neutrophils can be observed in the interstitium. Degeneration and focal necrosis with neutrophil infiltration were observed in hepatocytes. These pathological results indicate that severe inflammatory reactions or “inflammatory storms” may occur in patients with severe new coronavirus pneumonia. Therefore, the application of glucocorticoids may inhibit the inflammatory response and reduce organ damage. Academician Nanshan Zhong's team retrospectively analyzed the data of 1,099 patients with new coronavirus pneumonia and suggested that 5% of the severe patients were admitted to the ICU, and the overall mortality was 1.4%. However, the hospitalized mortality of severe patients was as high as 8.1%, and the proportion of severe patients using hormones was significantly higher than that of non-severe patients (44.5 vs. 13.7%) (11). Another observational study of patients with severe new coronavirus pneumonia showed that the 28-day mortality was as high as 61.5%, and patients who died were more likely to have ARDS than surviving patients (81 vs. 45%). Fifty-eight percent of patients were treated with combined hormone therapy and the survivors used hormones more often than the patients who died (70 vs. 50%) (12). In a retrospective analysis of 138 patients with new coronavirus pneumonia, 36 (26.1%) severe patients had a mortality rate of 16.6%, and the proportion of severe patients treated with glucocorticoids was significantly higher than that of non-severe patients (72.2 vs. 35.3%) (13). Clinicians are more inclined to use glucocorticoids for patients with severe new coronavirus pneumonia. The eighth editions of the “New Coronavirus Diagnosis and Treatment Program” (14) and “Shanghai Expert Consensus on Comprehensive Treatment of Coronavirus Diseases in 2019” (15) both recommend cautious limited use of glucocorticoids; they do not recommend routine use. For patients with acute exacerbation of dyspnoea, progressive deterioration of the oxygenation index and rapid progression on chest imaging, glucocorticoids (equivalent to methylprednisolone 1–2 mg/kg body weight/day, or 40–80 mg/day) can be used for a short period (3–5 days) as appropriate, and it should be noted that large doses of glucocorticoids will delay virus clearance due to immunosuppression.

## Experience in the Application of Glucocorticoids in the Treatment of Severe New Coronavirus Pneumonia

Our critical care team is involved in treating patients with severe new coronavirus pneumonia in the isolated ICU of the Shanghai public health clinical center, where critically ill patients require mechanical ventilation support, continuous blood purification, and even extracorporeal membrane oxygenation support. In the process of treating patients, we also face the following: (1) whether to use glucocorticoids in combination; (2) how much glucocorticoid should be used and for how long. In the following, we will provide a preliminary summary of the application of glucocorticoids in severe new coronavirus pneumonia based on the actual clinical diagnosis and treatment, previous ARDS drug treatment program, and literature evidence. Written informed consent was obtained from the [individual(s) AND/OR minor(s)' legal guardian/next of kin] for the publication of any potentially identifiable images or data included in this article. In addition, our retrospective observational case report was approved by the ethics committee of the relevant institution.

Patients with severe new coronavirus pneumonia often experience sudden exacerbation and a rapid progression of hypoxemia. Even if the patient is treated with non-invasive or invasive respiratory support in time, it is difficult for them to quickly improve their respiratory distress and hypoxia. At this time, the application of drugs must be considered for a comprehensive treatment. In addition to applying appropriate sedative and analgesic drugs to reduce oxygen consumption to adapt to the state of insufficient oxygen supply, it is also necessary to decide whether to use glucocorticoids and, if so, the dosage to use.

A 62-year-old female patient with a history of hypertension had been taking oral nifedipine tablets daily for a long time to control her blood pressure. She had no history of respiratory or immune system diseases. She was admitted to the hospital because of a “3-day fever.” She returned to Shanghai from Wuhan 16 days before admission. Her fever started 3 days before admission, and her condition deteriorated sharply. On admission, chest CT showed multiple patches of increased density in the right lung, and the new coronavirus nucleic acid sample was positive. The patient was given high-flow oxygen therapy to improve oxygenation, but her hypoxemia rapidly deteriorated within 10 h. The oxygenation index continued to decrease from ~200 to 60 mmHg. Under the condition of 60 L of oxygen flow and FiO_2_ = 0.9, her SpO_2_ was barely maintained at ~90%. The patient's heart rate and blood pressure increased, and oxygen consumption also increased significantly. In this case, in addition to non-invasive face-mask mechanical ventilation support and appropriate analgesia and sedation, methylprednisolone was given intravenously 40 mg every 12 h, while antibiotics were used to cover possible pathogenic bacteria, especially fungi. The patient's symptoms were notably relieved after 24–48 h, and the oxygenation index also increased to 150–180 mmHg. Meanwhile, the lymphocyte counts, which had been reduced to ~0.35 × 10^9^/L, and CD4+ cell counts, which had been reduced to ~100 cells/μL, were only slightly decreased. The methylprednisolone dose of 80 mg/day was changed to 40 mg/day after 5 days and then discontinued after 3 days. The patient was transferred out of the ICU 12 days after being admitted and is currently discharged. The lung CT in Figure 1 shows that the lung inflammation in this patient was significantly reduced after glucocorticoid treatment.

**Figure 1:** After glucocorticoid therapy, chest CT showed a significant decrease in the exudation of both lungs, suggesting decreased pulmonary inflammation.

Another patient was a 75-year-old male. He had a history of premature heart beats, no history of hypertension, and no history of respiratory or immune system diseases. There was also no clear history of travel to the epidemic area or exposure to the new coronavirus. Fever with shortness of breath and chest tightness appeared 10 days prior to admission. On admission, a CT scan of the chest showed extensive inflammation of both lungs, and SARS-CoV-2 infection was confirmed by a coronavirus nucleic acid test. Endotracheal intubation was given on the day of admission. The patients were given methylprednisolone at 40 mg every 12 h from admission. The dosage was reduced to 40 mg QD after 5 days and then stopped after 3 days. Tracheotomy was performed seven days after intubation. The patient's condition improved briefly after the first glucocorticoid treatment, but haemodynamic instability occurred suddenly, and lung compliance further decreased. The patient received ECMO support 7 days after tracheostomy ventilator support. At this point, the chest radiograph showed increased exudation of both lungs, and SpO_2_ could only be maintained at 85–88% under ECMO with a 4.5 L flow rate. Due to the patient's persistent candidiasis and poor control with amphotericin B, it was necessary to consider whether the rapid deterioration of the disease was caused by the exacerbation of infection (including fungus, G-bacilli and G+ cocci mixed infection) leading to septic shock or aggravation of coronavirus pneumonia. We adjusted the analgesic and sedative drugs and added muscle relaxants to reduce oxygen consumption while giving enhanced anti-infective treatment (posaconazole and meropenem). In addition, methylprednisolone was still administered intravenously at 40 mg every 12 h for 3 days after ECMO support; the dosage was changed to 40 mg QD after 3 days and then stopped 2 days later. On the day of deterioration, the follow-up examination showed that IL-6 increased from 735 to 4,212 pg/ml, and the lymphocyte count decreased from 2.83 × 109/L to 0.94 × 109/L. After 24–48 h of treatment, the vital signs of the patient stabilized, and SpO_2_ was maintained at ~95%. Additionally, IL-6 decreased to 289 pg/ml, the lymphocyte count decreased to 0.45 × 10^9^/L, and the CD4+ cell count decreased from 429 to 227 cells/μl. The above examination indicators showed a downward trend. However, at the same time, the blood culture continued to be positive for Candida, and retest with the fecal new coronavirus nucleic acid test was positive and continued to be strongly positive over the next few days. The chest radiograph of the patient showed that pulmonary inflammation did not improve significantly after glucocorticoid therapy (Figure 2). This patient died 5 weeks after ECMO support.

**Figure 2:** After glucocorticoid therapy, chest radiographs showed no significant reduction in pulmonary exudation, suggesting no improvement in lung inflammation.

In the first case, we found that early use of small doses of glucocorticoid was helpful for the improvement of the disease. In the second case, the cause of death may be that the prolonged use of glucocorticoids resulted in immunosuppression and serious fungal infections. In our experience, there were also a few patients whose condition had deteriorated sharply, with severe pulmonary exudation and marked systemic oedema accompanied by increased abdominal pressure. On the 1st day of deterioration, a large dose of 0.5 g of methylprednisolone was used, followed by 240 mg on the 2nd day. The patients' critical condition was significantly relieved after 48 h, but severe lymphocyte reduction and secondary fungemia appeared, which made subsequent treatment difficult. A recent study (16) found that in hospitalized patients with SARS-CoV-2, the use of dexamethasone resulted in lower 28-day mortality among those who were receiving either invasive mechanical ventilation or oxygen alone at randomization but did not result in lower 28-day mortality among those receiving no respiratory support. We believe that glucocorticosteroids can be used for the treatment of patients with SARS-CoV-2, but different therapeutic outcomes occur depending on the patient's underlying disease; comorbidities; severity of corona virus pneumonia; and type, timing, and dose of hormones used. Therefore, we are cautious about the use of glucocorticosteroids in the treatment of patients with SARS-CoV-2.

## Discussion

Our perspectives about glucocorticoid treatment is just based on the pharmacological characteristics of glucocorticoids and a small number of clinical cases, which is premature and need to be validated. Nevertheless, we are currently following the opinions, doses and timing of glucocorticoid application suggested in the Chinese Health Commission's recommendations (14, 15) during the process of diagnosis and treatment of severe new coronavirus pneumonia, and we have also observed some short-term effects in clinical practice. However, whether the long-term prognosis is improved requires further observation and research. The timing, dose, and type of glucocorticoid use, and even the patient's underlying conditions and comorbidities, also require stratified studies in multiple research centers with large sample sizes. In addition, it is noteworthy that although severe SARS-CoV-2 patients may experience excessive inflammation, they often suffer from severe cellular immune impairment (lymphocyte and CD4+ cell counts are significantly reduced). The application of glucocorticoids may further inhibit cellular immunity and delay virus clearance. Therefore, it is necessary to pay close attention to the possibility of fungal infections and perform a relevant culture. Prophylactic antifungal agents may be considered in critically ill patients to prevent the development of severe invasive fungal infections. Moreover, it is also well-known that the use of corticosteroids may also activate a previous underlying infection, such as hepatitis B virus or tuberculosis.

Glucocorticoids work by suppressing the abnormal immune response that destroys the body's organs rather than attacking the virus. In the case of new coronavirus pneumonia, the abnormal immune response seems to be more damaging than the replication of the virus in the body. The patient's age, underlying disease, comorbidities, severity of new coronavirus pneumonia, and timing and dosage of glucocorticoids used can all influence the effectiveness of treatment. Whether patients benefit from glucocorticoid therapy “depends on choosing the right dose at the right time, in the right patient.”

## Data Availability Statement

The original contributions generated for the study are included in the article/supplementary material, further inquiries can be directed to the corresponding author/s.

## Ethics Statement

The studies involving human participants were reviewed and approved by the ethics committee of Shanghai sixth people's hospital. The patients/participants provided their written informed consent to participate in this study.

## Author Contributions

All authors listed have made a substantial, direct and intellectual contribution to the work, and approved it for publication.

## Conflict of Interest

The authors declare that the research was conducted in the absence of any commercial or financial relationships that could be construed as a potential conflict of interest.
